# Determining factors affecting the perceived usability of air pollution detection mobile application “AirVisual” in Thailand: A structural equation model forest classifier approach

**DOI:** 10.1016/j.heliyon.2022.e12538

**Published:** 2022-12-22

**Authors:** Ardvin Kester S. Ong, Yogi Tri Prasetyo, Poonyawat Kusonwattana, Klint Allen Mariñas, Nattakit Yuduang, Thanatorn Chuenyindee, Kirstien Paola E. Robas, Satria Fadil Persada, Reny Nadlifatin

**Affiliations:** a School of Industrial Engineering and Engineering Management, Mapúa University, 658 Muralla St., Intramuros, Manila 1002, Philippines; b International Program in Engineering for Bachelor, Yuan Ze University, 135 Yuan-Tung Road, Chung-Li 32003, Taiwan; c Department of Industrial Engineering and Management, Yuan Ze University, 135 Yuan-Tung Road, Chung-Li 32003, Taiwan; d Department of Industrial Engineering, Faculty of Engineering, North-Chiang Mai University, Chiang Mai 50230, Thailand; e Department of Industrial and Systems Engineering, Chung Yuan Christian University, Taoyuan 320, Taiwan; f Department of Industrial Engineering and Aviation Management, Navaminda Kasatriyadhiraj Royal Air Force Academy, Bangkok, 10220, Thailand; g Entrepreneurship Department, BINUS Business School Undergraduate Program, Bina Nusantara University, Jakarta 11480, Indonesia; h Department of Information Systems, Institut Teknologi Sepuluh Nopember, Kampus ITS Sukolilo, Surabaya 60111, Indonesia

**Keywords:** Air pollution, Perceived usability, Protection motivation theory, System usability

## Abstract

Air pollution has been evident worldwide. It presented numerous pieces of evidence that affect health-related adverse effects causing diseases and even death and the development of technology has helped monitor the exposure of people to air pollution. This research analyzed factors affecting the perceived usability of air pollution detection on the ‘AirVisual’ mobile application based on the integrated model of Protection Motivation Theory (PMT) and Unified Theory of Acceptance and Use of Technology (UTAUT2). A total of 416 participants voluntarily answered a self-administered survey consisting of adapted constructs covering factors such as Performance expectancy (PE), Effort expectancy (EE), Social influence (SI), Facilitating conditions (FC), Habit (HB), Perceived risk (PR), Perceived trust (PT), Intention to use (IU), and Perceived usability (PU). Structural Equation Modeling and Random Forest Classifier were utilized to determine factors affecting perceived usability of the ‘AirVisual’ mobile application. The results showed that PE, EE, SI, and FC were key factors leading to very high PU among users. Moreover, IU was seen to be the most significant factor affecting PU, followed by PT, PR, and HB. This study is one of the first studies that considered the evaluation of usability among health-related mobile applications covering air pollution. The results and the framework utilized in this model may be applied to evaluate other factors and applications related to health among people. Lastly, this study can also be extended to evaluate other mobile applications worldwide.

## 1 Introduction

Air pollution is one of the most crucial issues in the world. It is the overview into the atmosphere of biological materials such as particulates, chemicals, and compounds that affect mental health, disease, even death to humans, plants, animals, and natural habitats (Balogun et al., 2021; Sarker, 2022; McDonald et al., 2020; Toro et al., 2021; Zhang et al., 2022). It has been considered one of the prominent environmental problems nowadays which has caused premature death worldwide. In 2019, a total of 4.2 million premature deaths were evident due to air pollution present outdoors (World Health Organization; Health Organization, 2022).

Usually, populated areas such as urban regions have been hotspots for carbon emissions. It was seen in Europe that around 85% of the population had been exposed to particulate matter (PM2.5) (von Schneidemesser et al., 2019). It was also seen in North America that several respiratory and cardiovascular diseases were present due to air pollution (Phosri et al., 2019). Phosri et al. (2019) explained how developing countries like those in the Asian Region have been reported to be exposed heavily to air pollution aside from developed countries like Western Europe. Takahashi et al. (2020) added that developing countries in Asia have been left underexplored when air pollution studies are taken into consideration. One of the countries that have experienced epidemiological evidence is Thailand.

Bangkok and metropolitan regions in Thailand are widely known as the most polluted area in the country which presented adverse health disease consequences. Vichi-Vadakan and Vajanapoom (2011) presented three major sources of air pollution in Thailand coming from vehicles using fossil fuel, forest or biomass burning, and industrial manufacturing allowing the release of carbon emissions to the surroundings. The growing air pollution of cities belongs to key problems coming from increased traffic, highly densely populated areas, high energy consumption, and lack of resources to monitor policy for sustainability.

With over 10 million people living in the capital of Thailand, Bangkok, transportation has been seen to be the main cause of several heavy particles present on roadsides (Mihăiţă et al., 2019). To which, Nitrogen Oxides (NO_2_), Sulfur Dioxide (SO_2_) and Carbon Monoxide/Dioxide (CO/CO_2_), and sources from vehicle exhaust have been heavily present since January 2007 (Paoin et al., 2021). The Pollution Control Department of Thailand has found PM2.5 present, exceeding the standard level yearly (Gebhart, 2016). It was explained that PM2.5 is not easily dispersed and would lead to accumulation that causes adverse health effects, especially in Thailand (Phosri et al., 2019). With that, the Thai government implemented several prevention measures to help mitigate the adverse health effects. One of those prevention measures is the development of the ‘AirVisual’ mobile application.

‘AirVisual’ is a mobile application (Figure 1) that provides air quality monitoring in Thailand. It partnered with the United Nations Environment Programme (UNEP) with programmers from Germany and Switzerland (Feenstra et al., 2019). This application is available on iOS and Android platforms which can be downloaded easily. It gathers data that could be accessed by individuals, companies, governments, and even different countries to measure the standard created by UNEP's global health policies. Available for 80 countries, this application has only been downloaded and installed by 241,265 mobile users from Google play and ranked 9th for the weather category in IOS. ‘AirVisual’ provides real-time air quality status (good, moderate, unhealthy) from your current place, nearby cities, and even major cities around the globe; it also provides your air pollution exposure and risks based on age groups. This shows the under the exploration of the beneficial mobile application worldwide. Since ‘AirVisual’ is developed for promoting a certain protection behavior using the mobile application, there are two theories that can be integrated to evaluate this mobile application, the Protection Motivation Theory and Unified Theory of Acceptance and Use of Technology.

**Figure 1:** ‘AirVisual’ mobile application.

Protection Motivation Theory (PMT) has been utilized to explain the understanding of fear and coping appraisal of people (Ong et al., 2021; Gumasing et al., 2022). PMT has been lengthened for more useful to reduce the threat and disease among individuals. This model has turned the behavior of people on the cognitive perspective to protect themselves (Prasetyo et al., 2020). In China, Ruan et al. (2020) utilized PMT to understand the behavior of tourists in air pollution. They presented that perceived risk, response, and self-efficacy had a significant effect on people's intentions. Moreover, the government response showed a significant and negative effect on behavioral intention. In Iran, Shafiei and Maleksaeidi (2020) presented how students possessed high response efficacy and environmental attitude through PMT towards pro-environmental behavior. Moreover, Janmaimool (2017) utilized PMT to evaluate the behavior of private and public office workers toward adverse consequences of pollutants. Their result showed that proper communication would lead to the engagement of people toward the mitigation of pollution. In relation to this study, the ‘AirVisual’ application was made available for anyone to use to enhance engagement. However, with the low scale of usage, the mobile application itself should be explored. To which, the Unified Theory of Acceptance and Use of Technology may be utilized to evaluate the technology at hand.

Unified Theory of Acceptance and Use of Technology (UTAUT2) is a theory that evolved from UTAUT (Venkatesh and Xu, 2012). This theory based on technology acceptance and usage has integrated several factors to consider the performance expectation, effort expectancy, social influence, and facilitation conditions, which can significantly affect the behavioral intention and acceptance of technology (Tamilmani et al., 2021). Tamilmani et al. (2021) explained how UTAUT2 is one of the highest-quality theories that could be utilized to evaluate the acceptance and use of any system or technology. Gansser and Reich (2021) utilized UTAUT2 to evaluate products with artificial intelligence integration for everyday life environments. Their result showed how mobility, household, and health were three segments taken into consideration for people to have behavioral intentions. Yuan et al. (2015) considered UTAUT2 to evaluate users’ perception of health and fitness applications. Their result presented that significant factors such as social influence, performance expectancy, and habit under UTAUT2 influences user continuous adoption in using the application.

Previously, several studies have dealt with mobile applications in regard to air pollution reduction. However, designs and assessments of air pollution were mostly developed. This shows how an available mobile application – an easily utilized air pollution monitoring technology has been underexplored. Yu et al. (2020) utilized mobile phone location data to evaluate people's exposure to CO_2_, NO_2_, SO_2_, Ozone (O_3_) at the ground level, and PM2.5. Their result showed that the information is not readily available and that it is difficult to warn people against the harmful pollutants available. Arku et al. (2018) developed an ultrasonic personal aerosol sampler to measure air pollution in households to monitor PM2.5. Their study characterized available air pollution and aimed to accurately estimate air pollution exposure. On the other hand, Zalakeviciute et al. (2019) generalized the evaluation of usability and accessibility function of available mobile applications for air pollution monitoring. They indicated that there is a need to explore more on the utility of the application since data and information are difficult to access (Zalakeviciute et al., 2019). This, therefore, reduces the knowledge available to the community. Thus, there is a need to assess easily accessible mobile applications such as ‘AirVisual’ to enhance the understanding and knowledge of the people, mitigate air pollution exposure, and create a positive behavioral intention to utilize the influential mobile application. In addition, Nyarku et al. (2018) presented mobile phone monitoring of individuals for air pollution exposure can be a major step in reducing health-related diseases.

This study aimed to identify relationships among the important factors of ‘AirVisual’ mobile application usability by integrating PMT and UTAUT2. Different latent variables such as performance expectancy, effort expectancy, social influence, facilitating conditions, habit, perceived risk, and perceived trust were evaluated to measure the intention to use and perceived usability of the ‘AirVisual’ mobile application. Utilizing Structural Equation Modeling (SEM) and Random Forest Classifier, the different factors were evaluated to identify the significant factors affecting the intention and perception of usability among users of the air pollution monitoring application. This study is one of the first studies that evaluated the mobile application that helps in mitigating air pollution. The result of this study could be utilized to help reduce air pollution proliferation by means of the promotion of ‘AirVisual’ usage in different countries. Finally, the integrated model can be applied and extended to evaluate other applications considering health-related factors worldwide.

## 2 Conceptual framework

The PMT and UTAUT2 frameworks were integrated into this study to measure the perceived usability of the ‘AirVisual’ mobile application. Figure 2 represents the conceptual framework utilized in this study. In this study, a total of 8 hypotheses were created for different latent variables under UTAUT2 including performance expectancy, effort expectancy, social influence, facilitating conditions, and habit. Moreover, latent variables under PMT include perceived risk and perceived trust. All these were hypothesized to have a significant effect on the intention to use, followed by perceived usability.

**Figure 2:** Conceptual framework.

Adapted from several studies, PMT is utilized to measure any coping and fear appraisal factors that may affect the health of an individual (Ong et al., 2021). Similarly, Gumasing et al. (2022) explained how the different factors under PMT may lead to the behavioral intention of people. On the other hand, UTAUT2 has been utilized to measure the acceptance and usage of technology (Venkatesh and Xu, 2012). Moreover, Tamilmani et al. (2021) systematically evaluated studies utilizing UTAUT2 and found that the dimensions considered in this theory can be considered to be of high quality for evaluating systems and technology usability. Thus, both theories were integrated to holistically measure a technology that affects an individual's health.

Venkatesh and Xu (2012) explained performance expectancy as the level of attaining the benefit from the system. The study of Zhang et al. (2019) presented a highly significant relationship between performance expectancy and intention among patients’ usage of diabetes management applications. The study of Cao and Niu (2019) resulted in performance expectancy as the only significant factor affecting user adaptation in a third-party payment platform. Moreover, Wang et al. (2003) expressed the significance of performance expectancy towards the intention of an individual to utilize technology. In the context of this study, since the application is being utilized for the benefit of health-related factors for an individual, then it was hypothesized that:

H1 Performance Expectancy has a significant effect on Intention to Use.

Effort expectancy is the level of ease of usage among individuals when using a system of technology (Venkatesh and Xu, 2012). Sharma et al. (2018) explained how effort expectancy is latent that is significant when determining intention and usage related to the ease of use of technology. Alalwan et al. (2017) and Lallmahomed et al. (2017) presented studies that showed how effort expectancy significantly affects the intention to use applications and systems among people. In addition, Palau-Saumell et al. (2019) showed how effort expectancy is a significant factor affecting the usage of mobile applications among consumers of food. Therefore, the ease of use of a system may be evaluated through effort expectancy and thus it was hypothesized that:

H2 Effort Expectancy has a significant effect on Intention to Use.

The people around an individual can cause either a positive or negative influence on them. To which, Min et al. (2019) showed how social influence can cause a significant effect on the intention to utilize transportation mobile applications. The compatibility and the people around an individual cause the positive influence to continuously utilize a mobile application. Campbell and Russo (2003) also explained how social context and interaction cause a significant relationship towards mobile usage. In this case, when people around an individual patronize the usage of the ‘AirVisual’ mobile application, it may present an present influence the individual to have the intention to use it also. Therefore, it was hypothesized that:

H3 Social Influence has a significant effect on Intention to Use.

Facilitating conditions are the level of support available for the usage of a system (Venkatesh and Xu, 2012). Lu et al. (2016) showed how facilitating conditions affect a person's intention to adopt wireless technology. In addition, Lallmahomed et al. (2017) presented a high significance between facilitating conditions and intention to use when the internet and the application are easily accessible. Moreover, Alalwan et al. (2017) showed how facilitating conditions would have a positive significant effect on an individual's intention to use technology when they perceive that the resources are available and easily accessible. Since ‘AirVisual’ application is available for mobile applications, it was hypothesized that:

H4 Facilitating Conditions has a significant effect on Intention to Use.

Habit is the development of an individual to continuously utilize a system or technology (Venkatesh and Xu, 2012). Okumus et al. (2018) explained how the availability of technology nowadays has been well adopted by people thus reducing the highlight of difficulty applying it in daily activities. Moreover, Lu et al. (2016b) presented how the positive mobility drive of an individual resulted in a positive intention to utilize mobile applications. In the context of this study, ‘AirVisual’ application has been widely utilized in Thailand after the event of air pollution is present in a certain location. Thus, it was hypothesized that:

H5 Habit has a significant effect on Intention to Use.

From the results of the study by Cao and Niu (2019), they presented how utilizing an application may present risk perception among users. It was explained that when people have a low perception of risks, they would have a positive intention to utilize a mobile application (Martins et al., 2014). Mingxing et al. (2014) showed how perceived risk and perceived trust are key indicators for users to have behavioral intention in utilizing mobile applications. In addition, it was explained in the study of Kapser and Abdelrahman (2020) that people consider the possible risk present in a system or technology before they utilize it. Therefore, trust among people should be built before individuals would positively patronize the utility of an application (Chuenyindee et al., 2022; Sharma et al., 2018; Prasetyo and Soliman, 2021; Lallmahomed et al., 2017). Lallmahomed et al. (2017) explained how trust perceived by an individual significantly affects their intention to use an application. To which, the following were hypothesized:

H6 Perceived Risk has a significant effect on Intention to Use.

H7 Perceived Trust has a significant effect on Intention to Use.

From the study of Gelderblom et al. (2019), they presented how perceived usability is highlighted when there is a positive intention to continuously use a system. Moreover, Pee et al. (2018) explored how there is a positive intention when there is high usability seen among users. This explained how the advantages of using an application are taken into consideration when assessing the usability and could be preceded by high intentions of usage. In addition, Fernandes et al. (2020) explained how the intention to use causes a positive influence on the perceived usability adopted from the system usability scale (SUS) assessment. Moreover, Mavlanova et al. (2012) relate website usability to customers’ intention to use it for grocery shoppers. The results of their study showed that when website usability caters to the users there will be a repeat order. Therefore, it was hypothesized that:

H8 Intention to Use has a significant effect on Perceived Usability.

## 3 Methodology

### 3.1 Respondents

A total of 416 Thais participated in this study, collected via convenience sampling. Presented in Table 1 is the descriptive statistics of the respondents from the metropolitan and provincial region in Bangkok that were affected by fine particulate matter (PM2.5). The participants considered in this study have installed and used the ‘AirVisual’ application on their mobile phones. The data were gathered from January to March 2021 when PM2.5 spread around Thailand. As seen in Table 1, 58.27% of the respondents were female while 40.78% were male around 25–34 years old (52.88%), 15–24 years old (15.38%), and 35–44 years old (14.18%). To which, the majority had 10,001–20,000 THB (23.56%) monthly salary/allowance, 20,001–30,000 THB (21.63%), and 15.87% had more than 50,000 THB. Moreover, most of the respondents had a Bachelor's degree (57.69%) and a Master's degree (24.52%). Lastly, 72.84% had health insurance and 27.16% had none. This study was approved by Mapua University Research Ethics Committees (FM-RC-21-55). Informed consent was obtained from all participants prior to the data collection.

**Table 1:** The demographic data of the respondents (n = 416).

Characteristics	Category	N	%
Gender	Male	170	40.78
	Female	242	58.27
	Other	4	0.95
Age	15–24	64	15.38
	25–34	220	52.88
	35–44	59	14.18
	45–54	40	9.62
	55–64	30	7.21
	More than 64	3	0.72
Income/Allowance per month	<10,000 THB	65	15.63
	10,001–20,000 THB	98	23.56
	20,001–30,000 THB	90	21.63
	30,001–40,000 THB	50	12.02
	40,001–50,000 THB	47	11.30
	More than 50,000 THB	66	15.87
Education	Secondary school certificate or below	4	0.96
	High school	15	3.61
	Diploma	22	5.29
	Bachelor's degree	240	57.69
	Master's degree	102	24.52
	Doctoral degree	30	7.21
	Other	3	0.72
Do you have Health insurance?	Yes	303	72.84
	No	113	27.16

### 3.2 Questionnaire

Table 2 represents the constructs utilized in the study. The measurement items were adapted from the UTAUT2 and PMT to measure which factors influenced with usability of the ‘AirVisual’ mobile application user (Gansser and Reich, 2021). Similarly, Gansser and Reich (2021) utilized and extended UTAUT2 to evaluate the acceptance of products such as mobility, household, and health with artificial intelligence (AI). Consequently, this study measured factors affecting intention to use and perceived usability of mobile applications. From the PMT, perceived risk and perceived trust were considered for the latent, adapted from several studies (Ong et al., 2021; Gefen et al., 2000). A total of 39 items were considered adapted and modified for measuring factors affecting the perceived usability of ‘AirVisual’ mobile application.

**Table 2:** Construction frameworks.

Constructs	Item	Measurement	References
Performance Expectancy	PE1	I found AirVisual mobile application is helpful in my daily life.	Venkatesh and Xu (2012)
	PE2	Using AirVisual mobile application to alert protecting danger from PM 2.5 increases health protection for me.	Gansser and Reich (2021)
	PE3	Using AirVisual mobile application helps me prepare and understand protection from PM 2.5 daily.	Gansser and Reich (2021)
	PE4	Using the AirVisual mobile application helps me achieve and prepare for health protection from PM 2.5 easier.	Gansser and Reich (2021)
	PE5	I found the system unnecessarily complex.	Venkatesh and Xu (2012)
Effort Expectancy	EE1	I expect AirVisual mobile application would be easy to use.	Venkatesh and Xu (2012)
	EE2	My interaction with the AirVisual mobile application is clear and understandable.	Venkatesh and Xu (2012)
	EE3	Learning how to use AirVisual mobile application alert of hazardous from PM 2.5 is easy for me.	Gansser and Reich (2021)
	EE4	It is easy for me to become an expert at using AirVisual mobile application.	Venkatesh and Xu (2012)
	EE5	I would imagine that most people would learn to use AirVisual very quickly.	Venkatesh and Xu (2012)
Social Influence	SI1	The important persons in my life think I should use the AirVisual mobile application.	Gansser and Reich (2021)
	SI2	The important person in my life who influences my behavior thinks I should use the AirVisual mobile application.	Gansser and Reich (2021)
	SI3	The important person in my life whose opinions I prefer influenced me to use AirVisual mobile application.	Gansser and Reich (2021)
	SI4	The important person in my life who uses the AirVisual mobile application makes my interested to use it.	Gansser and Reich (2021)
Facilitating Conditions	FC1	I have the necessary tools to use the AirVisual mobile application.	Alalwan et al. (2017)
	FC2	I would expect to have the necessary knowledge to use the AirVisual mobile application.	Venkatesh and Xu (2012)
	FC3	The AirVisual mobile application is applicable with my mobile phone.	Alalwan et al. (2017)
	FC4	I would be able to get help from other people when I have difficulties using the AirVisual mobile application.	Alalwan et al. (2017)
Habit	HB1	Using AirVisual mobile application is easy.	Prasetyo et al. (2021a)
	HB2	Using AirVisual mobile application is enjoyable.	Prasetyo et al. (2021a)
	HB3	Using AirVisual mobile application is entertaining.	Prasetyo et al. (2021a)
	HB4	Using AirVisual mobile application is secure.	Prasetyo et al. (2021a)
Perceived Risk	PR1	Using AirVisual mobile application to alert hazards of PM2.5 would still have the risk.	Ong et al. (2021)
	PR2	Using AirVisual mobile application to alert hazard of PM2.5 would remind me of air pollution risk.	Ong et al. (2021)
	PR3	Using AirVisual mobile application to alert hazardous PM2.5 is helping to decrease my health risk.	Ong et al. (2021)
	PR4	Using AirVisual mobile application to alert hazard of PM2.5 is increasing my knowledge of health risk from air pollution.	Ong et al. (2021)
Perceived Trust	PT1	I believe the AirVisual mobile application is trustworthy when it comes to updates.	Gefen and Straub (2003)
	PT2	Even if not monitored, I may trust the AirVisual mobile application to do work properly.	Alalwan et al. (2017)
	PT3	I believe the Air Quality Index in the AirVisual mobile application is accurate.	Gefen and Straub (2003)
	PT4	I am assured with the technological sufficiency to protect me from PM2.5 air pollution problems on the AirVisual mobile application.	Alalwan et al. (2017)
Intention to use AirVisual application	IU1	I intend to use the AirVisual mobile application in the future.	Prasetyo et al. (2021a)
	IU2	I would always try to use the AirVisual mobile application in my daily life when available.	Prasetyo et al. (2021a)
	IU3	I would always install the AirVisual mobile application on my mobile phone when I change my mobile phone in the future.	(Chuenyindee et al., 2022); (Ong et al., 2022)
	IU4	I plan to use the AirVisual mobile application for checking air quality index when I see the weather is different (presence of fog).	
Perceived Usability	PU1	I found the AirVisual mobile application very comfortable to use.	Sonderegger and Sauer (2010)
	PU2	I found the air Quality Index in the AirVisual mobile application is working well and was well consolidated.	Sonderegger and Sauer (2010)
	PU3	I found the air quality index on the AirVisual mobile application is easy to understand.	Sonderegger and Sauer (2010)
	PU4	I take a little time to understand all of the functions of the AirVisual mobile application.	Sonderegger and Sauer (2010)
	PU5	I think AirVisual mobile application is a useful mobile application	Sonderegger and Sauer (2010)

### 3.3 Structural Equation Modeling

IBM Analysis of Moment Structures (AMOS) 24 was utilized to develop the Structural Equation Modeling (SEM) considered in this study. The causal relationships between each latent variable were measured using SEM (Gumasing et al., 2023; Hair, 2010). Similar to previous studies, SEM was utilized to evaluate the usage behavior of individuals. Jun et al. (2019) considered the integration of UTAUT2 and PMT to evaluate the initial adoption and use intention of advanced driver assistance (ADAS). To which, their study developed a diffusion and marketing strategy for ADAS. Duarte and Pinho (2019) considered SEM to evaluate mobile health adoption among people from Portugal. Their result suggested that combining with another tool would result in a more comprehensive result towards the SEM insignificant latent. In addition, Fan et al. (2016) explained how the SEM may consider some latent to be insignificant due to the indirect effects present in the model. In addition, this study employed Random Forest Classifier as another tool to verify the contributing factors affecting the perceived usability of ‘AirVisual’ mobile application.

### 3.4 Random Forest Classifier

Random Forest Classifier (RFC) is a machine learning algorithm that considers the classification of different factors affecting human behavior (Chen et al., 2019)(Yuduang et al., 2022). Gao et al. (2021) presented how RFC may be a viable tool for predicting factors that results in higher accuracy. Moreover, considering RFC produces the best split and branch among other decision trees present (Snehil and Goel, 2020). Thus, this study considered RFC using Python 4.5. Specifically, data cleaning was employed using correlation analysis. Only p-values less than 0.05 and correlation coefficient greater than 0.20 were considered significant.

A total of 16,224 datasets was considered in the algorithm as every indicator was deemed significant. After data normalization, the RFC optimization considered a total of 6,400 runs employing different parameters to obtain the optimum tree. Parameters such as the splitter (gini or entropy), criterion (best or random), training and testing ratios (60:40–90:10), and tree depth (4–7) were considered with 100 runs for each combination.

## 4 Results

### 4.1 Structural Equation Modeling

Figure 3 represents the initial SEM for factors affecting perceived usability for ‘AirVisual’ mobile application. As seen from the model, FC4 has a factor loading below the threshold of 0.5 (Hair, 2010). With that, this construct was removed. Moreover, performance expectancy and social influence had p-values greater than 0.05. To which, these latent variables were removed as well and the model was run to generate the final SEM.

**Figure 3:** The initial SEM model of AirVisual.

Presented in Figure 4 is the final model for factors affecting perceived usability of ‘AirVisual’ mobile application. Out of 8 hypotheses, only 6 were accepted from the SEM result. Modification indices were performed to enhance the model fit of the study (Prasetyo et al., 2021a). Presented in Table 3 are the descriptive statistics of the constructs together with the final factor loading considered in this study.

**Figure 4:** The final SEM model of Factors Affecting the Perceived Usability of Air Pollution Detection Mobile Application “AirVisual”.

**Table 3:** Descriptive statistics and validity.

Latent Variables	Items	Mean	StD	Cronbach's α	Factor Loadings	Average Variance Extracted (AVE)	Composite Reliability (CR)
	FC1	4.1442	0.89355	0.788	0.798	0.557	0.790
Facilitating Conditions	FC2	4.1683	0.84486		0.718		
	FC3	4.3221	0.76495		0.721		
	HB1	4.2380	0.79976		0.774		
HB	HB2	3.6418	1.01748	0.765	0.891	0.564	0.835
	HB3	3.2380	1.20585		0.727		
	HB4	4.0192	0.89152		0.580		
	PR1	4.0000	0.95438	0.725	0.657	0.522	0.813
Perceived Risk	PR2	4.2428	0.82794		0.721		
	PR3	4.0986	0.88216		0.722		
	PR4	4.1418	0.88988		0.784		
	PT1	3.8413	0.89109	0.886	0.856	0.668	0.890
Perceived Trust	PT2	3.8534	0.88093		0.799		
	PT3	3.8654	0.86771		0.868		
	PT4	3.7356	0.95553		0.739		
	EE1	4.3774	0.76007		0.570		
	EE2	4.1803	0.83230		0.777		
Effort Expectancy	EE3	4.2115	0.79666	0.851	0.854	0.543	0.854
	EE4	4.0697	0.85444		0.753		
	EE5	4.1130	0.82095		0.699		
	PU1	4.2139	0.80054	0.909	0.819	0.611	0.887
	PU2	4.0409	0.82477		0.772		
Perceived Usability	PU3	4.1947	0.80843		0.804		
	PU4	4.1731	0.82072		0.724		
	PU5	4.2909	0.77895		0.786		
	IU1	4.2644	0.81391	0.912	0.820	0.634	0.873
Intention to Use	IU2	4.2548	0.84024		0.825		
	IU3	4.1587	0.87472		0.818		
	IU4	4.2596	0.84734		0.716		

Based on the results, it could be seen that all constructs had values greater than the threshold, 0.5. Moreover, Ong et al. (2021b) explained how Cronbach's alpha and the Composite Reliability should have values greater than 0.7 while the average variance extracted should be greater than 0.5. This would present internal validity and reliability for the final model created (Hair, 2010). Table 4 presents the model fit considered in this study. Following the suggestion of Gefen et al. (2000), GFI and AGFI could have values greater than 0.80 while IFI, TLI, and CFI could have a minimum of 0.9 to indicate the model has an acceptable fit (Hair, 2010). Moreover, the RMSEA value should have less than 0.07. Thus, the final model is considered to be acceptable.

**Table 4:** Model fit.

Goodness of fit measures of the SEM	Parameter Estimates	Minimum cut-off	Recommended by
Goodness of Fit Index (GFI)	0.859	>0.80	Gefen et al. (2000)
Adjusted Goodness of Fit Index (AGFI)	0.863	>0.80	Gefen et al. (2000)
Root Mean Square Error of Approximation (RMSEA)	0.065	<0.07	Hair (2010)
Incremental Fit Index (IFI)	0.919	>0.90	Hair (2010)
Tucker Lewis Index (TLI)	0.925	>0.90	Hair (2010)
Comparative Fit Index (CFI)	0.938	>0.90	Hair (2010)

Performing Harman's Single Factor Test for Common Method Bias (CMB), the constructs presented a result equal to 16.967%. Ong et al. (2021b) explained how values less than 50% present no CMB. Moreover, the Shapiro-Wilks test was done to determine the normality. The result presented values within the threshold of ±1.96. Thus, no CMB is present and the data is normally distributed. Presented in Table 5 is the causal relationship of the latent considered in this study.

**Table 5:** Fornell-Larcker criterion.

Factor	EE	FC	HB	PR	PT	IU	PU
EE	0.737						
FC	0.644	0.746					
HB	0.542	0.697	0.75				
PR	0.603	0.591	0.511	0.722			
PT	0.491	0.618	0.667	0.572	0.817		
IU	0.538	0.692	0.509	0.604	0.616	0.796	
PU	0.705	0.684	0.609	0.598	0.638	0.733	0.782

For further testing of results, discriminant validity using Fornell-Larcker Criterion (FLC) and Heterotrait-Monotrait (HTMT) Ratio was conducted. Presented in Table 5 is the Fornell-Larcker Criterion. Based on the findings, the diagonal values are much greater compared to the values in the horizontal and vertical results. It was indicated by Ong et al. (2021b) and Hair (2010) that this presents a valid dataset.

In addition, the HTMT Ratio was conducted as presented in Table 6. Following the suggestion of Kline (2018), a 0.85 threshold was set to have an acceptable HTMT value. In addition, Rahman et al. (2018) indicated a 0.90 threshold for HTMT values. From the results, all are lower than 0.85 which indicates – together with the FLC, how the results and dataset utilized are valid. In addition, presented in Table 7 are the causal relationships of the latent considered in this study.

**Table 6:** HTMT ratio.

Factors	EE	FC	HB	PR	PT	IU
FC	0.656					
HB	0.845	0.806				
PR	0.831	0.835	0.782			
PT	0.756	0.668	0.571	0.82		
IU	0.641	0.686	0.843	0.689	0.834	
PU	0.65	0.779	0.7	0.795	0.843	0.781

**Table 7:** Direct, indirect, and total effects.

No	Variable	Direct Effect	P-Value	Indirect Effect	P-Value	Total Effect	P-Value
1	PT → IU	0.429	0.005	–	–	0.429	0.005
2	PR → IU	0.222	0.015	–	–	0.222	0.015
3	HB → IU	−0.120	0.043	–	–	−0.120	0.043
4	FC → IU	0.746	0.005	–	–	0.746	0.005
5	EE → IU	0.152	0.032	–	–	0.152	0.032
6	IU → PU	0.820	0.036	–	–	0.820	0.036
7	PT → PU	–	–	0.352	0.004	0.352	0.004
8	PR → PU	–	–	0.182	0.011	0.182	0.011
9	HB → PU	–	–	−0.098	0.037	−0.098	0.037
10	FC → PU	–	–	0.612	0.010	0.612	0.010
29	EE → PU	–	–	0.124	0.030	0.124	0.030

### 4.2 Random Forest Classifier

Following the suggestion of Duarte and Pinho (2019), another tool may be utilized to determine the most significant variable affecting the goal of the study. To which, this study considered employing RFC. After performing the optimization process, an analysis of variance (ANOVA) was conducted to determine the difference between the result of this study. Presented in Table 8 is the summarized result from the highest obtained average accuracy.

**Table 8:** Decision tree mean accuracy (depth = 5).

Category	60:40	70:30	80:20	90:10
Random				
**Gini**	86.70	94.00	90.90	92.50
**Std. Dev**	10.86	3.559	3.635	2.635
**Entropy**	91.50	94.90	93.40	93.00
**Std. Dev**	6.468	2.644	2.221	3.496
**Best**				
**Gini**	91.30	91.30	93.40	93.50
**Std. Dev**	0.949	1.159	0.843	2.415
**Entropy**	92.00	92.00	**95.00**	94.50
**Std. Dev**	0.000	0.000	**0.000**	0.581

The ANOVA presented no significant difference among the results obtained. To which, this study considered the tree from the results with the highest average accuracy of 95% and with 0.000 standard deviations. The optimum tree considered was with entropy as the splitter, best criterion, 80:20 training and testing ratio, and depth equal to 5. Figure 5 represents the optimum tree considered for the classification of factors affecting the perceived usability of ‘AirVisual’ mobile application.

**Figure 5:** Optimum tree from random forest classifier (depth = 5).

Based on the result, effort expectancy (X1) is the parent node that would lead to considering a value less than or equal to 0.312. If satisfied, this will consider social influence (X2) which will lead to very high perceived usability and facilitating condition (X3) if not. X2 will consider X3 if this is will not satisfied which will lead to X1 and very high perceived usability if satisfied. However, it will consider performance expectancy (X0) if not satisfied which will lead to very high perceived usability when satisfied for values less than or equal to 0.05. When the condition of X3 from the second node will be satisfied, it will consider X1 which will lead to very high perceived usability for ‘AirVisual’ mobile application. Thus, it could be deduced that the main factors affecting perceived usability for ‘AirVisual’ mobile application are performance and effort expectancy, social influence, and facilitating conditions.

## 5 Discussion

This study integrated UTAUT2 and PMT to determine factors affecting the perceived usability of the air pollution detection mobile application, ‘AirVisual’ in Thailand. To evaluate, SEM and RFC were employed to classify the different factors considered in this study such as Performance Expectancy (PE), Effort Expectancy (EE), Social Influence (SI), Facilitating Conditions (FC), Habit (HB), Perceived Risk (PR), Perceived Trust (PT), Intention to Use (IU), and Perceived Usefulness (PU).

Based on the RFC results, EE would be the parent node indicating that this factor would be the most significant factor affecting the perceived usability of ‘AirVisual’ mobile application. This was also a significant latent from the SEM result on IU (β: 0.152, p = 0.032). Based on the indicator, people find the application easy to use, clear and understandable, and quick even for other people to use. Like any other mobile application, there should be less effort and quick navigation for them to continuously utilize it. A similar discussion was present in the study by Sharma et al. (2018). Their study discussed how less effort in utilizing the mobile application would enhance an individual's IU. Different studies also presented EE as a significant factor affecting IU (Alalwan et al., 2017; Lallmahomed et al., 2017; Prasetyo et al., 2021b). This justifies why there is an indirect effect of EE on PU (β: 0.125, p = 0.030).

Second, SI was considered a significant factor for RFC but was deemed insignificant for SEM. Woody (2011) presented challenges for the results of SEM if a full mediation variable was considered in a model. Employing the suggestion of Duarte and Pinho (2019), another tool may be considered to evaluate the significance of the latent from SEM. This justifies why RFC considered SI still as a significant latent. SI indicators include important people around them influence usage. Usually, people around us influence our motivation to utilize an application (Ahmad and Khalid, 2017). Similarly, Palau-Saumell et al. (2019) explained how the perception of people around an individual influences their IU when everyone is utilizing a mobile application. Consequently, different studies (Palau-Saumell et al., 2019; Sharma et al., 2018) also integrated different tools with SEM and resulting in SI being a significant factor. Generally, it was explained that the current generation is already well adapted to the advancement of mobile technology, thus reducing the SI on people's IU.

Third, FC was considered as a significant latent for both RFC and second-highest from SEM (β: 0.746, p = 0.005). The constructs presented that people have the necessary tools and knowledge to use the application, easy usage for mobile phones and it is easy to ask for help when something is not understood from the application. FC is the ease of utility with a system or technology being considered. Lallmahomed et al. (2017) presented how FC is latent with a high relationship with IU due to the availability of the internet and application for people to use. This supports the indirect effect of FC on PU (β: 0.612, p = 0.010). It was explained that people pay attention to available resources for them to utilize that would be beneficial in their daily lives (Sharma et al., 2018; Alalwan et al., 2017).

In addition, the RFC considered PE as a significant factor however very low value was considered. Subsequently, SEM presented that this latent was not significant. Following the suggestion of Fan et al. (2016), this may be due to the presence of a mediator considered in this study. From the constructs, it could be deduced that ‘AirVisual’ is helpful daily, alert to protect from PM2.5, and helps protect and prepare for PM2.5. PE is the degree of benefits obtained by individuals upon using a specific system or application (Palau-Saumell et al., 2019; Venkatesh and Xu, 2012). Based on the construct, it could be referred to that ‘AirVisual’ is important with health-related benefits to individuals in Thailand. Venkatesh and Xu (2012) and Wang et al. (2003) established that PE is a core latent in measuring the intention of an individual to utilize a system or technology. In relation to this study, it provides protection and information for preparation against harmful PM2.5.

Continuing with the SEM results, the highest significant factor affecting PU was IU (β: 0.820, p = 0.036). It presents that people will continue using the application even in the future, apply the usage of the application daily, install the application when changing mobile phones, and use the application for checking the air quality when there is unusual fog present. This posits that people have seen the benefit towards health benefits of using the mobile application against air pollution. This entails them continuously utilizing the ‘AirVisual’ mobile application. Gelderblom et al. (2019) explained how IU could be highlighted when there is positive usability on a certain system of technology. In addition, Pee et al. (2018) explored website usability and intention to repurchase. It was highlighted that when people see the advantages of utilizing a certain application, there would be continuous usage, highlighting also trust built among users.

PT was also seen to have a direct significant effect on IU (β: 0.429, p = 0.005) and an indirect effect on PU (β: 0.352, p = 0.004). Indicators of PT show that the application is trustworthy for air pollution updates, no monitoring is needed since the application notifies automatically, with high accuracy, and assured that the technology can protect from PM2.5 pollution among people. Based on the experience of people, it could be inferred that trust in the information provided by the mobile application was evident. Moreover, it was seen that information provided was deemed accurate. Similar to the findings by Merhi et al. (2019), it was found that trust has a direct significant effect on behavioral intention in terms of mobile banking. Similarly, Pee et al. (2018) explained that users’ trust should be built upon continuous patronage of utility. Moreover, Sharma et al. (2018) and Lallmahomed et al. (2017) presented trust as one of the most significant latent affecting adoption and usability.

Moreover, PR was considered to have a direct significant effect on IU (β: 0.222, p = 0.015) and an indirect effect on PU (β: 0.182, p = 0.011). From the indicators, ‘AirVisual’ can send alerts during hazardous PM2.5 presence, send reminders of pollution risks, and increase knowledge of pollution risk present. Thus, utilizing the application can reduce health risks as well. This implies that with frequent notifications and alerts, the risk of air pollution effects among people has been reduced. The key importance of reducing the risk of air pollution was seen as apparent with the ‘AirVisual’ mobile application. Kapser and Abdelrahman (2020) found that PR influences IU, wherein users prefer to know the risk of the service provided before they can consider perceiving it as something useful. In the context of this study, Thais were able to see the benefits of health-related factors upon utilizing the ‘AirVisual’ mobile application. Ong et al. (2021) explained how knowing the benefit would highlight people's acceptance of a specific matter. In this case, the intention to continuously use the mobile application due to the reduced risk of PM2.5.

Interestingly, HB had a negative direct significant effect on IU (β: −0.120, p = 0.042) and an indirect effect on PU (β: −0.098, p = 0.037). This presents that the application is not that easy to use, not enjoyable, not entertaining, and may have questionable security. These deferred the habit to become negative in terms of using ‘AirVisual’ mobile application. Palau-Saumell et al. (2019) explained how this is a key factor affecting IU. However, Okumus et al. (2018) explained how the availability of technology nowadays has been well adopted by people thus reducing the highlight of difficulty in applying it in daily activities. This shows that people have the capabilities to consider this as part of their daily activity without too much effort. Thus, it explains why people would continuously utilize the ‘AirVisual’ mobile application despite the results of this study as they see the benefit and advantages towards their health and daily lives.

Overall, people find comfort in using the ‘AirVisual’ mobile application in their daily lives. It could be deduced that the application was well consolidated and is working well. Moreover, there is moderate ease of use present from the mobile application, there is little time needed to understand the information present, and the mobile application is a useful tool to help prepare for air pollution.

### 5.1 Theoretical contribution

This research applied several theoretical to the existing literature on PMT and UTAUT2. First, this research provided the significant factors affecting the perceived usability of the ‘AirVisual’ mobile application, especially during the period of air pollution problems in Thailand. Based on the results, it could be deduced that the factors under UTAUT2 go beyond measuring the perceived usability of the mobile application. Rather, it was seen from the results that even with negative habits seen, people will continuously utilize an application as long as their health is being considered. This presents that the key importance of a system could be highlighted based on the constant information update (PE), less effort in navigation (EE), more people utilizing the application (SI), and beneficial for daily lives (FC) would lead to a positive intention to use the application which is deemed very high perceived usability among people.

Moreover, when health-related factors are taken into consideration, then the integration of PMT could be referred to as one of the most important theoretical frameworks that could be considered. Both the coping appraisal and threat appraisal factors could be considered to measure the intention of an individual. When trust (coping) and risk (threat) has been established, then it could help evaluate why people would have the continuous motivation to utilize the application at hand. Thus, it could be stated that the integration of both UTAUT2 and PMT holistically measures why a health-related mobile application may be patronized by people.

Lastly, the consideration of machine learning algorithms such as RFC towards the assessment of factors affecting a certain subject aside from SEM has been deemed beneficial. It could be seen that the limitation of using only SEM has been evident due to the available mediating effect or the indirect effect present from the integrated model. The consideration of integrated tools in assessing factors of human behavior is beneficial to evaluate the results and findings of a study.

### 5.2 Practical implications

This study presented how the ‘AirVisual’ mobile application developed and utilized in Thailand has been seen as beneficial among people. As air pollution cannot be measured and seen by the naked eye, automated tracing and updates are required so people would know when and how to protect themselves when this event is relatively high. The finding of this study can be used as a guideline to improve the mobile application. Based on the result, people are using the application due to the benefit it has towards health-related factors. However, it was seen that it is not easy, enjoyable, entertaining, and security may be questionable. Thus, it is suggested that developers may enhance the system so people to easily use the application.

There has been a positive result showing that people will still continue using the application in the future, even plans to download the application when they change mobile phones. The developer of the application may take advantage of this finding to continuously promote the patronage of the ‘AirVisual’ application. In addition, they may also promote the application by highlighting how health-related benefits could be seen when using the application. It was found that there is a positive effect when people know and see the benefit of the ‘AirVisual’ application. Thus, these factors may be considered to garner more users for the mobile application which would be beneficial for the people and developers as well. The findings of this study could also be considered by other countries to monitor the air quality present, which will help people to prepare and mitigate any pollution available worldwide.

### 5.3 Limitations and future research

This research acknowledges several limitations despite sufficient findings. First, this study only considered respondents with experience in using the ‘AirVisual’ application. The people who answered the self-administered survey have already practiced and gained knowledge of how the mobile application is being utilized. It may be beneficial to consider responses among people with first and no experience at using the application to highlight factors affecting their intention to use and perceived usability. Second, due to the COVID-19 pandemic, this study only considered a self-administered survey. This has been a limit since the established framework was considered to build the adapted constructs for the study. Interviews may be conducted to highlight other factors that affect people's perceptions and intentions. Moreover, more factors may be developed for the extension of the integrated framework after the evaluation of the interview. Lastly, this study considered only RFC as the machine learning algorithm. Despite the high average accuracy obtained for this study, other machine learning algorithms may be considered such as neural networks with SEM to consider the most significant factor affecting intention to use and perceived usability. In addition, clustering of respondents may be done to indicate which demographics consider the factors considered in this study.

## 6 Conclusion

Air pollution has been considered one of the serious problems present globally. In Thailand, the presence of air pollution from years ago still affects the current generation. Problems regarding the respiratory tract and other health-related problems are still evident. To which, Thais utilize the ‘AirVisual’ mobile application to help reduce and mitigate air pollution if present in an area.

This study utilized the Protection Motivation Theory (PMT) integrated with Unified Theory of Acceptance and Use of Technology (UTAUT2) to identify the factors affecting the perceived usability of air pollution detection mobile application, ‘AirVisual’. This was measured among Thai people who were affected by air pollution. A total of 416 participants voluntarily answered a self-administered survey analyzed using Structural Equation Modeling (SEM) and Random Forest Classifier (RFC). The result from RFC showed that Effort Expectancy (EE), Social Influence, Facilitating Conditions (FC), and Performance Expectancy were factors that would lead to very high Perceived Usefulness (PU). Based on the result from SEM, Intention to Use was the highest significant factor affecting PU, followed by FC, Perceived Trust, Perceived Risk, and EE. It was seen that Habit had a negative direct effect on PU.

It was seen that people would highlight more on the benefits and advantages when health-related factors against air pollution are being considered. Despite the difficulty of using the application, the benefits were seen to overpower the challenges of using the mobile application. The results and findings of this study could be applied and extended by other developers to create a similar application for air pollution monitoring worldwide. Moreover, the benefit of having this type of mobile application may reduce the risk of people towards exposed to air pollution. Finally, this study can be applied to use in other fields related to protection motivation and hazard with other mobile applications (Khaw et al., 2022) (Al-Emran et al., 2020, Al-Emran et al., 2022, Campbell and Russo, 2003, Snehil and Goel, 2020).

## Declarations

### Author contribution statement

Ardvin Kester S. Ong, Ph.D.; Yogi Tri Prasetyo, Ph.D.; Poonyawat Kusonwattana, Ph.D.; Klint Allen Mariñas, Ph.D. Candidate: Conceived and designed the experiments; Performed the experiments; Analyzed and interpreted the data.

Contributed reagents, materials, analysis tools or data; Wrote the paper.

Nattakit Yuduang, Ph.D.; Thanatorn Chuenyindee, Ph.D.; Kirstien Paola E. Robas, BS Industrial Engineering; Satria Fadil Persada, Ph.D.; Reny Nadlifatin, Ph.D.: Analyzed and interpreted the data; Contributed reagents, materials, analysis tools or data.

### Funding statement

This research did not receive any specific grant from funding agencies in the public, commercial, or not-for-profit sectors.

### Data availability statement

Data will be made available on request.

### Declaration of interest's statement

The authors declare no competing interests.

### Additional information

No additional information is available for this paper.

## References

[bib1] Ahmad S.Z., Khalid K. (2017). The adoption of M-government services from the user’s perspectives: empirical evidence from the United Arab Emirates. Int. J. Inf. Manag..

[bib2] Alalwan A.A., Dwivedi Y.K., Rana N.P. (2017). Factors influencing adoption of mobile banking by Jordanian Bank customers: extending UTAUT2 with trust. Int. J. Inf. Manag..

[bib3] Al-Emran M., Granić A., Al-Sharafi M.A., Ameen N., Sarrab M. (2020). Examining the roles of students' beliefs and security concerns for using smartwatches in higher education. J. Enterprise Inf. Manag..

[bib4] Al-Emran M., Al-Nuaimi M.N., Arpaci I., Al-Sharafi M.A., Anthony B. (2022). Towards a wearable education: understanding the determinants affecting students' adoption of wearable technologies using machine learning algorithms – education and Information Technologies. SpringerLink.

[bib5] Arku R.E., Birch A., Shupler M., Yusuf S., Hystad P., Brauer M. (2018). Characterizing exposure to household air pollution within the prospective urban rural epidemiology (PURE) study. Environ. Int..

[bib6] Balogun A.-L., Tella A., Baloo L., Adebisi N. (2021). A review of the inter-correlation of climate change, air pollution and urban sustainability using novel machine learning algorithms and Spatial Information Science. Urban Clim..

[bib7] Campbell S.W., Russo T.C. (2003). The cocial construction of mobile telephony: an application of the social influence model to perceptions and uses of mobile phones within personal communication networks. Commun. Monogr..

[bib8] Cao Q., Niu X. (2019). Integrating context-awareness and Utaut to explain Alipay user adoption. Int. J. Ind. Ergon..

[bib9] Chen J., Li Q., Wang H., Deng M. (2019). A machine learning ensemble approach based on random forest and radial basis function neural network for risk evaluation of regional flood disaster: a case study of the Yangtze river delta, China. Int. J. Environ. Res. Publ. Health.

[bib71] Chuenyindee T., Montenegro L.D., Ong A.K., Prasetyo Y.T., Nadlifatin R., Ayuwati I.D., Sittiwatethanasiri T., Robas K.P. (2022). The perceived usability of the learning management system during the COVID-19 pandemic: Integrating System Usability Scale, technology acceptance model, and task-technology fit. Work.

[bib75] Chuenyindee T., Ong A.K., Prasetyo Y.T., Persada S.F., Nadlifatin R., Sittiwatethanasiri T. (2022). Factors affecting the perceived usability of the COVID-19 contact-tracing application “Thai chana” during the early COVID-19 omicron period. International Journal of Environmental Research and Public Health.

[bib67] Duarte P., Pinho J.C. (2019). A mixed methods UTAUT2-based approach to assess mobile health adoption. Journal of Business Research.

[bib10] Fan Y., Chen J., Shirkey G., John R., Wu S.R., Park H., Shao C. (2016). Applications of structural equation modeling (SEM) in Ecological Studies: an updated review. Ecol. Processes.

[bib11] Feenstra B., Papapostolou V., Hasheminassab S., Zhang H., Boghossian B.D., Cocker D., Polidori A. (2019). Performance evaluation of twelve low-cost PM2.5 sensors at an ambient air monitoring site. Atmos. Environ..

[bib12] Fernandes J., Teles A., Teixeira S. (2020). An augmented reality-based mobile application facilitates the learning about the spinal cord. Educ. Sci..

[bib13] Gansser O.A., Reich C.S. (2021). A new acceptance model for artificial intelligence with extensions to UTAUT2: an empirical study in three segments of application. Technol. Soc..

[bib14] Gao G., Li Z., Huan Z., Chen Y., Liang J., Zhou B., Dong C. (2021). Human behavior recognition model based on feature and classifier selection. Sensors.

[bib15] Gebhart G. (2016). https://asiafoundation.org/2014/03/26/transboundary-pollution-in-northern-thailand-causes-dangerous-levels-of-smog/.

[bib16] Gefen D., Straub D., Boudreau M. (2000). Structural equation modeling and regression: guidelines for research practice. Commun. Assoc. Inf. Syst..

[bib17] Gefen Karahanna, Straub (2003). Trust and tam in online shopping: an integrated model. MIS Q..

[bib18] Gelderblom H., Matthee M., Hattingh M., Weilbach L. (2019). High school learners’ continuance intention to use electronic textbooks: a usability study. Educ. Inf. Technol..

[bib19] Gumasing M.J., Prasetyo Y.T., Ong A.K., Nadlifatin R. (2022). Determination of factors affecting the response efficacy of Filipinos under Typhoon Conson 2021 (jolina): an extended protection motivation theory approach. Int. J. Disaster Risk Reduc..

[bib72] Gumasing M.J., Prasetyo Y.T., Ong A.K., Persada S.F., Nadlifatin R. (2023). Factors influencing the perceived usability of wearable chair exoskeleton with market segmentation: A structural equation modeling and K-means clustering approach. International Journal of Industrial Ergonomics.

[bib20] Hair J.F. (2010).

[bib21] Janmaimool P. (2017). Application of protection motivation theory to investigate sustainable waste management behaviors. Sustainability.

[bib66] Jun, J., Park, H., & Cho, I. (2019). Study on initial adoption of Advanced Driver Assistance System: Integrated Model of PMT and utaut 2. *Total Quality Management & Business Excellence*, *30*(sup1).

[bib22] Kapser S., Abdelrahman M. (2020). Acceptance of autonomous delivery vehicles for last-mile delivery in Germany – extending UTAUT2 with risk perceptions. Transport. Res. C Emerg. Technol..

[bib23] Khaw K.W., Alnoor A., Al-Abrrow H., Chew X.Y., Sadaa A.M., Abbas S., Khattak Z.Z. (2022). Modelling and evaluating trust in mobile commerce: a hybrid three stage fuzzy Delphi, structural equation modeling, and neural network approach. Int. J. Hum. Comput. Interact..

[bib24] Kline R.B. (2018). Response to Leslie Hayduk’s review of principles and practice of structural equation modeling, 4th edition. Can. Stud. Popul..

[bib25] Lallmahomed M.Z.I., Lallmahomed N., Lallmahomed G.M. (2017). Factors influencing the adoption of e-government services in Mauritius. Telematics Inf..

[bib26] Lu J., Yu C., Chang L. (2016). Facilitating conditions, wireless trust and adoption intention. J. Comput. Inf. Syst..

[bib27] Lu J., Liu C., Wei J. (2016). How important are enjoyment and mobility for mobile applications?. J. Comput. Inf. Syst..

[bib28] Mavlanova T., Benbunan-Fich R., Koufaris M. (2012). Signaling theory and information asymmetry in online commerce. Inf. Manag..

[bib29] Martins C., Oliveira T., Popovič A. (2014). Understanding the internet banking adoption: a unified theory of acceptance and use of technology and Perceived Risk Application. Int. J. Inf. Manag..

[bib30] McDonald F., Horwell C.J., Wecker R., Dominelli L., Loh M., Kamanyire R., Ugarte C. (2020). Facemask use for community protection from Air Pollution Disasters: an ethical overview and framework to guide agency decision making. Int. J. Disaster Risk Reduc..

[bib31] Merhi M., Hone K., Tarhini A. (2019). A cross-cultural study of the intention to use mobile banking between Lebanese and British consumers: extending UTAUT2 with security, Privacy and Trust. Technol. Soc..

[bib32] Mihăiţă A.S., Dupont L., Chery O., Camargo M., Cai C. (2019). Evaluating air quality by combining stationary, Smart Mobile Pollution Monitoring and data-driven modelling. J. Clean. Prod..

[bib33] Min S., So K.K.F., Jeong M. (2019). Consumer adoption of the Uber mobile application: insights from diffusion of innovation theory and technology acceptance model. J. Trav. Tourism Market..

[bib34] Mingxing S., Jing F., Yafang L. (2014). 2014 International Conference on Cyber-Enabled Distributed Computing and Knowledge Discovery.

[bib35] Nyarku M., Mazaheri M., Jayaratne R., Dunbabin M., Rahman M.M., Uhde E., Morawska L. (2018). Mobile phones as monitors of personal exposure to air pollution: is this the future?. PLoS One.

[bib36] Okumus B., Ali F., Bilgihan A., Ozturk A.B. (2018). Psychological factors influencing customers’ acceptance of smartphone diet apps when ordering food at restaurants. Int. J. Hospit. Manag..

[bib37] Ong A.K., Prasetyo Y.T., Salazar J.M., Erfe J.J., Abella A.A., Young M.N., Chuenyindee T., Nadlifatin R., Ngurah Perwira Redi A.A. (2021). Investigating the acceptance of the reopening Bataan nuclear power plant: integrating protection motivation theory and extended theory of planned behavior. Nucl. Eng. Technol..

[bib38] Ong A.K., Prasetyo Y.T., Lagura F.C., Ramos R.N., Sigua K.M., Villas J.A., Young M.N., Diaz J.F., Persada S.F., Redi A.A. (2021). Factors affecting intention to prepare for mitigation of “The big one” earthquake in the Philippines: integrating protection motivation theory and extended theory of planned behavior. Int. J. Disaster Risk Reduc..

[bib73] Ong A.K., Prasetyo Y.T., Yuduang N., Nadlifatin R., Persada S.F., Robas K.P., Chuenyindee T., Buaphiban T. (2022). Utilization of random forest classifier and artificial neural network for predicting factors influencing the perceived usability of COVID-19 contact tracing “Morchana” in Thailand. International Journal of Environmental Research and Public Health.

[bib39] Palau-Saumell R., Forgas-Coll S., Sánchez-García J., Robres E. (2019). User acceptance of mobile apps for restaurants: an expanded and extended utaut-2. Sustainability.

[bib40] Paoin K., Ueda K., Ingviya T., Buya S., Phosri A., Seposo X.T., Seubsman S.-ang, Kelly M., Sleigh A., Honda A., Takano H., Chokhanapitak J., Churewong C., Hounthasarn S., Khamman S., Pandee D., Pangsap S., Prapamontol T., Puengson J. (2021). Long-term air pollution exposure and self-reported morbidity: a longitudinal analysis from the Thai Cohort Study (TCS). Environ. Res..

[bib41] Pee L.G., Jiang J., Klein G. (2018). Signaling effect of website usability on repurchase intention. Int. J. Inf. Manag..

[bib42] Phosri A., Ueda K., Phung V.L., Tawatsupa B., Honda A., Takano H. (2019). Effects of ambient air pollution on daily hospital admissions for respiratory and cardiovascular diseases in Bangkok, Thailand. Sci. Total Environ..

[bib43] Prasetyo Y.T., Castillo A.M., Salonga L.J., Sia J.A., Seneta J.A. (2020). Factors affecting perceived effectiveness of COVID-19 prevention measures among Filipinos during enhanced community quarantine in Luzon, Philippines: integrating Protection Motivation Theory and extended theory of planned behavior. Int. J. Infect. Dis..

[bib76] Prasetyo, Y. T., & Soliman, K. O.(2021). Usability evaluation of ERP systems: A comparison between SAP S/4 Hana & Oracle Cloud. 2021 IEEE 8th International Conference on Industrial Engineering and Applications (ICIEA)

[bib44] Prasetyo Y.T., Tanto H., Mariyanto M., Hanjaya C., Young M.N., Persada S.F., Redi A.A. (2021). Factors affecting customer satisfaction and loyalty in online food delivery service during the COVID-19 pandemic: its relation with open innovation. J. Open Innov.: Technol., Market, Complexity.

[bib45] Prasetyo Y.T., Ong A.K., Concepcion G.K., Navata F.M., Robles R.A., Tomagos I.J., Young M.N., Diaz J.F., Nadlifatin R., Redi A.A. (2021). Determining factors affecting acceptance of e-learning platforms during the COVID-19 pandemic: integrating Extended Technology Acceptance Model and Delone & McLean is success model. Sustainability.

[bib46] Rahman M.M., Adedeji S.B., Bashir M.A., Islam J., Reaz M., Khan A.M. (2018). Mediation using covariance based-structural equation modeling (CB-SEM): the why and how?. Asian J. Empir. Res..

[bib47] Ruan W., Kang S., Song H.J. (2020). Applying protection motivation theory to understand international tourists’ behavioural intentions under the threat of Air Pollution: a Case of Beijing, China. Curr. Issues Tourism.

[bib48] Sarker M.S. (2022). Assessing levels of migrant-friendliness in the context of vulnerability to climate variability, change and environmental hazard: a comparison of two different-sized cities. Int. J. Disaster Risk Reduc..

[bib49] Shafiei A., Maleksaeidi H. (2020). Pro-environmental behavior of university students: application of Protection Motivation theory. Global Ecol. Conserv..

[bib50] Sharma S.K., Al-Badi A., Rana N.P., Al-Azizi L. (2018). Mobile applications in Government Services (MG-app) from user's perspectives: a predictive modelling approach. Govern. Inf. Q..

[bib51] Snehil, Goel R. (2020). Flood damage analysis using machine learning techniques. Procedia Comput. Sci..

[bib52] Sonderegger A., Sauer J. (2010). The influence of design aesthetics in usability testing: effects on user performance and perceived usability. Appl. Ergon..

[bib53] Takahashi M., Feng Z., Mikhailova T.A., Kalugina O.V., Shergina O.V., Afanasieva L.V., Heng R.K., Majid N.M., Sase H. (2020). Air pollution monitoring and tree and forest decline in east Asia: a review. Sci. Total Environ..

[bib54] Tamilmani K., Rana N.P., Wamba S.F., Dwivedi R. (2021). The extended unified theory of acceptance and use of Technology (UTAUT2): a systematic literature review and theory evaluation. Int. J. Inf. Manag..

[bib55] Toro A.,R., Catalán F., Urdanivia F.R., Rojas J.P., Manzano C.A., Seguel R., Gallardo L., Osses M., Pantoja N., Leiva-Guzman M.A. (2021). Air pollution and covid-19 lockdown in a large South American city: santiago Metropolitan Area, Chile. Urban Clim..

[bib56] Venkatesh Thong, Xu (2012). Consumer acceptance and use of information technology: extending the unified theory of acceptance and use of Technology. MIS Q..

[bib57] Vichit-Vadakan N., Vajanapoom N. (2011). Health impact from air pollution in Thailand: current and future challenges. Environ. Health Perspect..

[bib58] von Schneidemesser E., Steinmar K., Weatherhead E.C., Bonn B., Gerwig H., Quedenau J. (2019). Air pollution at human scales in an urban environment: impact of local environment and vehicles on particle number concentrations. Sci. Total Environ..

[bib59] Wang Y.S., Wang Y.M., Lin H.H., Tang T.I. (2003). Determinants of user acceptance of internet banking: an empirical study. Int. J. Serv. Ind. Manag..

[bib60] Woody E. (2011). An SEM perspective on evaluating mediation: what every clinical researcher needs to know. J. Exp. Psychopathol..

[bib70] World Health Organization. (2022). *Ambient (outdoor) Air Pollution*. World Health Organization. Retrieved December 23, 2022, from https://www.who.int/news-room/fact-sheets/detail/ambient-(outdoor)-air-quality-and-health

[bib61] Yu X., Ivey C., Huang Z., Gurram S., Sivaraman V., Shen H., Eluru N., Hasan S., Henneman L., Shi G., Zhang H., Yu H., Zheng J. (2020). Quantifying the impact of daily mobility on errors in air pollution exposure estimation using mobile phone location data. Environ. Int..

[bib62] Yuan S., Ma W., Kanthawala S., Peng W. (2015). Keep using my health apps: discover users' perception of health and fitness apps with the UTAUT2 model. Telemed. e-Health.

[bib74] Yuduang N., Ong A.K., Vista N.B., Prasetyo Y.T., Nadlifatin R., Persada S.F., Gumasing M.J., German J.D., Robas K.P., Chuenyindee T., Buaphiban T. (2022). Utilizing structural equation modeling–artificial neural network hybrid approach in determining factors affecting perceived usability of mobile mental health application in the Philippines. International Journal of Environmental Research and Public Health.

[bib63] Zalakeviciute R., Alexandrino K., Acosta-Vargas P., Pérez-Medina J.-L., Hernandez W. (2019). Evaluation of smart phone open source applications for Air Pollution. Adv. Intell. Syst. Comput..

[bib64] Zhang Y., Liu C., Luo S., Xie Y., Liu F., Li X., Zhou Z. (2019). Factors influencing patients’ intentions to use diabetes management apps based on an extended unified theory of acceptance and use of technology model: web-based survey. J. Med. Internet Res..

[bib65] Zhang G., Ren Y., Yu Y., Zhang L. (2022). The impact of air pollution on individual subjective well-being: evidence from China. J. Clean. Prod..

